# A Single-Center Treatment Experience of Gamma Knife Radiosurgery for Optic Pathway Glioma

**DOI:** 10.1155/2022/2043515

**Published:** 2022-08-09

**Authors:** Youlin Ge, Zhiyuan Zhang, Yanhe Li, Yiguang Lin, Yongqing Zong, Dong Liu

**Affiliations:** Department of Gamma Knife Center, The Second Hospital of Tianjin Medical University, Tianjin, China

## Abstract

**Objectives:**

To determine the independent prognostic factors that will influence the local tumor control/visual acuity (VA) preservation of optic pathway glioma (OPG) after Gamma Knife radiosurgery (GKS) and to optimize the treatment strategy.

**Methods:**

A cohort of 52 consecutive OPG patients who underwent GKS in our center between August 1997 and September 2020 was studied retrospectively. Risk factors such as age at GKS, gender, tumor subtype, tumor site, tumor volume, intratumoral cyst formation, and marginal dose were selected for the univariate and multivariate analysis. COX proportional hazard models were built to determine the independent prognostic factors of local tumor control/VA preservation, and the Kaplan-Meier (K-M) curves were plotted to compare the survival rate among subgroups.

**Results:**

52 OPG patients were included in this study, with a median age of 13.8 years (2-53 years); female outnumbered male at a ratio of 30 : 22; 7 patients (13.5%) had a history of surgical resection; 14 patients (26.9%) were categorized as neurofibromatosis type I (NFI) associated OPG and the rest as sporadic OPG; there were 6 patients (11.5%) with tumors located at hypothalamus/optic chiasm and the rest located in the orbit; the mean tumor volume was 4.36 ml (0.25-11.4 ml); 49 patients (94.2%) presented with VA impairment before GKS; 28 patients (53.8%) underwent single fraction GKS, and the rest underwent fractionated GKS (2-4 fractions); the mean marginal dose (represented with biologically effective dose, BED) was 66.6 Gy (13.3-126.0 Gy); the median follow-up time was 39 months (6-147 months); 11 patients were observed with tumor relapse, 33 with stable disease, and 8 with tumor regression; tumor relapse time varied from 30 to 76 months (mean 54 months); the 1-, 3-, and 5-year progression-free survival (PFS) rates were 100%, 92%, and 78%, respectively; 30 patients were included in the visual analysis; 7 patients were observed with VA deterioration, 19 with stable VA, and 4 with VA improvement; the 1-,3-, and 5-year VA preservation rates were 92%, 84%, and 77%, respectively. COX proportional hazard risk models showed that intratumoral cyst formation and marginal dose were the only two independent prognostic factors of local tumor control/VA preservation; fractionated GKS provided a higher VA preservation rate than single fraction GKS. Four patients were observed with conjunctive edema/conjunctive hyperemia in 1-4 weeks after GKS.

**Conclusions:**

GKS is a safe and effective treatment for OPG either as initial treatment or as salvage treatment after surgical resection, it provides good local tumor control and VA preservation, and fractionated GKS could be a preference for OPG patients with baseline VA ≥ 0.2.

## 1. Introduction

Optic pathway glioma (OPG) is one of the most common optic neurogenic tumors, especially in childhood, and it arises from any site of the optic pathway, mainly the orbit and the optic chiasm/hypothalamus. According to the presentation, OPG is categorized to NFI-associated OPG and sporadic OPG; the former often occurs in children and the latter often in adults. OPG patients usually present with VA impairment, proptosis, strabismus, headache, etc.; furthermore, OPG at optic chiasm/hypothalamus can lead to precocious puberty or stunting in children. Unfortunately, there is no standard therapy for OPG; until now, chemotherapy, radiotherapy, and surgery remain the mainstay for OPG treatment. Chemotherapy is often considered as the initial treatment of OPG in some previous studies; cisplatin and vincristine are widely used as the first-line regimens [1]; in recent years, novel therapies such as selumetinib [2] and bevacizumab [3] are used for the treatment of OPG. Surgical resection of OPG is a big challenge for neurosurgeons, constricted to the adjacent vital structures such as optic nerve, optic chiasm, or hypothalamus; resection is usually accompanied with a high rate of morbidity and mortality [4]; occasionally, resection or biopsy is performed for the purpose of histopathological diagnosis in pediatric OPG. Radiotherapy is usually carried out after chemotherapy or surgical resection as an adjuvant or salvage therapy, but when to initiate radiothrapy remains controversial; in the past few decades, stereotactic radiosurgery/radiotherapy was widely used for the treatment of OPG and achieved favorable outcomes in local tumor control and VA preservation; now, it is usually selected as the initial treatment for pediatric OPG. We treated more than eighty OPG patients with GKS from August 1997 to September 2020 in our center and retrospectively studied the outcome to determine the independent prognostic factors of local tumor control and VA preservation.

## 2. Methods and Materials

### 2.1. Patient Selection

Fifty-two out of eighty-four consecutive OPG patients were included in this study; the inclusion criteria are as follows: (1) patients diagnosed as NFI-associated/sporadic OPG approved by histopathology or radiological findings; (2) patients who underwent GKS as initial/adjuvant/salvage treatment in our center; (3) with a follow-up time ≥ 6 months, including visual and radiological follow-up; and (4) with detailed medical documentations (in-patient and out-patient). Patients who died of other diseases or followed up ≤6 months were excluded. On MRI images, OPG typically appeared as tubular or fusiform in shape that surrounds the optic nerve or optic chiasm, isointense on T1-weighted images, and iso-/hyperintense on T2-weighted images; after administration of gadolinium, the lesion appears uniform enhancement; if there are intratumoral cysts, OPG appears mixed hyperintense [5]. This study was approved by the Institutional Review Board of Tianjin Medical University.

### 2.2. GKS Procedure

The GKS treatment group is composed of a neurosurgeon, a radiation oncologist, a neurologist, and a radiation physicist. The GKS procedure starts with fixing the rigid stereotactic frame (Leksell Model G) to the head of patients under local anesthesia, and then, a thin-slice (2 mm slice with no gap) brain magnetic resonance image (MRI) scan with standard T1- and T2-weighted and gadolinium contrast-enhanced images in axial and coronal plane is performed. If patients are contraindicated for gadolinium, a iohexol contrast-enhanced brain computed tomography (CT) is performed instead. Thereafter, the images are input into the GammaPlan Station 4.0, the tumor and organs at risk (OARs) are contoured before dose planning, and then, an appropriate marginal dose with a flexible isodose line is planned by the radiation oncologist to surround the tumor and ensure that the radiation exposure to the OARs is safe. Then, the patient is fixed on the automatic position system (APS) and carried out the dose plan; finally, the stereotactic frame is taken off when the treatment is finished. Glucocorticoid is administered intravenously after GKS to prevent radiation edema. The treatment units used in our center were Gamma Knife models B, C, and Perfexion in sequence. In recent years, we carried out fractionated GKS in some patients to prevent VA or OAR damage.

### 2.3. Follow-Up

Patients were scheduled to follow up in our center every half year in the first two years after GKS and annually thereafter if the outcomes were satisfactory. Clinical follow-up and radiological follow-up were performed simultaneously. Clinical follow-up was performed by another neurosurgeon in our center who did not participate in the GKS procedure; he/she mainly evaluated the evolution of patients' symptoms and signs and to determine if a further intervention was necessary. Radiological follow-up included brain MRI or CT scans, the images were downloaded and analyzed with ImageJ (Version 1.8), and the three longest diameters (head-tail diameter, anterior-posterior diameter, and transverse diameter) of tumors were measured, and tumor volume was calculated with the formulaV (ml) = head‐tail diameter × anterior‐posterior diameter × transverse diameter × *π*/6. Tumor response was described as complete response (CR), major response (MAR), partial response (PR), minor response (MIR), stable disease (SD), and progressive disease (PD) according to the Response Assessment in Pediatric Neuro-Oncology (RAPNO) [6]. VA measurement was performed independently by three members in our group, whether we used logMAR charts or key picture test depending on the age of subjects [7]. Since the visual data was somewhat subjective, we take the mean value of the three measurements as patients' VA to minimize the deviation.

We defined tumor relapse (PD) as the primary endpoint and vision loss ≥ 0.2 compared with baseline VA in the affected eyes as the secondary endpoint. Follow-up time was defined as the interval from the completion of GKS to the endpoint or the latest follow-up.

### 2.4. Data Statistics and Analysis

All treatment and follow-up data was collected from the GKS to the latest follow-up. Continuous data was described by mean (normal data) or median (nonnormal data), and categorical data was described by frequency and percentage for further analysis and statistics. We imputed the missing data by multiple random imputation. Marginal dose was represented with biologically effective dose (BED) in univariate and multivariate analyses.

Student's *T*-test was used for the comparison of normal data and chi-square test for the comparison of categorical data. K-M curves with log-rank test were plotted to show the difference of survival rates among subgroups. Patients' age, gender, tumor site, tumor volume, intratumoral cyst formation, marginal dose, etc., were selected for univariate analysis, variables with a *p* value < 0.15 entered the multivariate analysis, COX proportional hazard models were built to determine the independent prognostic factors, a *p* value < 0.05 was considered statistically significant, and the results were visualized with forest-plots. All data analysis and statistics were completed with R language (version 4.02).

## 3. Results

### 3.1. Demographic Characteristics

This cohort was composed of 52 OPG patients who underwent GKS and followed up in our center, including 42 pediatric OPG patients and 10 adult OPG patients. The median age at GKS was 13.8 years (2-53years); females outnumbered males at a ratio of 30 : 22; natural history of disease varied from 1 to 72 months; 7 patients (13.5%) experienced at least one surgical resection or biopsy before GKS; the diagnosis was approved by histopathology; the rest were diagnosed based on radiological findings and typical presentations [8]. No patients had chemotherapy or radiotherapy history before GKS. 14 patients (26.9%) were categorized to NFI-associated OPG and the rest as sporadic OPG. All patients were found with solitary OPG along the optic pathway, 46 OPGs (88.5%) located in the orbit, and the rest located at the optic chiasm/hypothalamus. Mean tumor volume at GKS was 4.36 ml (0.25-11.4 ml). 42 tumors (80.8%) appeared as fusiform in shape, in which 10 tumors (19.2%) with intratumoral cyst. 49 patients (94.2%) presented with VA impairment, and 27 patients (51.9%) presented with ipsilateral proptosis. Other symptoms such as headache, orbital pain, and strabismus were rarely observed (Table 1).

### 3.2. GKS Procedure Parameters

Individualized GKS treatment strategies were applied to different OPG patients according to tumor site, tumor volume, adjacent OARs, and patients' expectation of VA. For patients with tumor ≥ 3 cm, or tumor involved the optic chiasm/hypothalamus, or baseline VA ≥ 0.2, fractionated GKS was scheduled to prevent the optic nerve or adjacent OARs damage, usually in 2-4 fractions; otherwise, single fraction GKS was performed. As a result, 28 (53.8%) patients underwent single fraction GKS (8.0-18.0 Gy), and the rest underwent fractionated GKS, in which 5 patients underwent two fractions GKS (7.0 Gy × 2), 12 patients underwent three fractions (6.0 Gy × 3), and 7 patients underwent four fractions (4.5 Gy × 4). Marginal physical dose was transformed to BED for further analysis and statistics; calculation of BED is [9]

(1) $$\begin{array}{c} \text{BED }\left(\text{Gy}\right)=D\left[1+\frac{d}{\alpha /\beta }\right], \end{array}$$

where *D* is the total physical dose, *d* is the physical dose per session, and *α*/*β* is the tissue-specific constant (Gy).

The marginal dose is represented with BED in the following sections. The prescription marginal dose varied from 26.7 to 126.0 Gy (mean 66.6 Gy). Given an overall physical dose, BED was negatively correlated with fractions in general; the more fractions, the smaller BED. The isodose lines varied from 45% to 70%; 8-26 isocenters were planned for each tumor.

### 3.3. Outcomes of Follow-Up

All patients included in this study were regularly followed for 6-147 months (median 39 months). Until the latest follow-up, 11 patients were observed with tumor relapse in 30-76 months (mean 54 months) after GKS, in which 8 patients with intraorbital OPG and the rest with optic chiasmatic/hypothalamic OPG; there were 7 patients in single fraction GKS group (28 patients) and 4 in fractionated GKS group (24 patients); the overall survival (OS) rate was 75.0% and 83.3%, respectively; the result was not statistically significant between two subgroups (chi-square test, *p* > 0.05); 5 patients were observed with tumor relapse and VA deterioration simultaneously. For further intervention, one patient with OPG located at the optic chiasm/hypothalamus underwent surgical resection, and the rest underwent a second GKS. 38 patients had stable disease, in which 2 patients experienced VA deterioration compared to the baseline VA. There were 3 patients with tumor shrinkage in 24-72 months after GKS (Figure 1). The 1-, 3-, and 5-year PFS rates of tumor control in this cohort were 100%, 92%, and 78%, respectively.

VA was measured independently by three members in our group, and we take the mean value of 3 measurements as the patients' VA. VA improvement/deterioration was defined as VA elevating/declining by 0.2 compared to the baseline VA. 22 patients with baseline VA < 0.2, in which 12 were blind in the affected eyes, were excluded for visual analysis, because this level of VA was considered unrecoverable and would eventually progress to blindness. For the rest 30 patients included in visual analysis, 4 patients were observed with VA improvement in 12-36 months after GKS, in which 3 patients were observed with SD and one with PR simultaneously; 19 patients were observed with stable VA after GKS, in which 16 patients were observed with SD and 3 with PD; the 1,-3-, and 5-year VA preservation rates were 92%, 84%, and 77%, respectively. Seven patients presented with VA deterioration in 6-36 months after GKS, in which 5 patients with single fraction GKS and 2 with fractionated GKS; the overall VA preservation rate was 68.8% and 85.7% in two subgroups, respectively; the result was not statistically significant (Fisher's test, *p* > 0.05) but clinically significant; it showed that fractionated GKS provided a higher VA preservation rate than single fraction GKS.

Four patients were observed with conjunctive edema/conjunctive hyperemia in 1-4 weeks after GKS and recovered after treated with eye drops; other side effect was rarely observed.

### 3.4. Data Analysis and Model Building

PFS was defined as the interval from GKS to the endpoint. Risk factors such as patients' age at GKS, gender, tumor site, intratumoral cyst formation, surgery history, tumor volume, and marginal dose were included in univariate analysis; continuous variables were split to subgroups according to the cutpoints of ROC plots. Factors with a *p* value ≤ 0.15 were considered clinically significant; as a result, tumor site, intratumoral cyst formation, tumor volume, and marginal dose were selected and entered the multivariate analysis; the differences of survival rate among subgroups were demonstrated with K-M curves (Figure 2). Multivariate COX proportional hazard model was built to determine the independent prognostic factors that impact the PFS; finally, intratumoral cyst formation and marginal dose (BED) were determined as the independent prognostic factors for local tumor control (Table 2); the result was visualized with forest-plot (Figure 3).

30 patients with baseline VA ≥ 0.2 were included in visual analysis; patients' age at GKS, subtypes of OPG (NFI-associated OPG and sporadic OPG), tumor site, intratumoral cyst formation, baseline VA, tumor volume, marginal dose (BED), etc., were selected for univariate analysis; the result is shown in Table 3. As a result, intratumoral cyst formation and marginal dose were selected and entered the multivariate analysis, although the *p* value of baseline VA and tumor volume was more than 0.15, but they were considered independent prognostic factors for VA preservation in some prior publications, so we also included them in the multivariate analysis; the differences of survival rate among subgroups were demonstrated with K-M curves (Figure 4). Finally, intratumoral cyst formation and marginal dose were determined as the independent prognostic factors for VA preservation according to the multivariate COX proportional hazard model (Table 3), and the result was visualized with forest-plot (Figure 5).

## 4. Discussion

### 4.1. Advances in OPG Treatment

OPG is a kind of low-grade glioma (LGG) that involves the optic pathway, which accounts for 2-5% of all central nervous system neoplasms. It is usually appears as pilocytic astrocytoma in histopathology (WHO grade I) [10]. According to the presentation, OPG is categorized to NFI-associated OPG and sporadic OPG; the former often occurs in children and the latter often in adults. NFI-associated OPG and sporadic OPG are different in genotype, presentation, and prognosis and require different treatment strategies consequently. Based on the fact that pediatric OPG is a self-healing disease in some children, if there is no VA impairment, patients are advised to follow up without any intervention, and the lesion often becomes indolent after puberty; once if there is vision damage, appropriate treatment should be recommended. Chemotherapy is the upfront therapy in many previous publications, cisplatin and vincristine are the first-line regimens for pediatric OPG, and the VA outcomes were proved satisfactory [11–13]. In recent years, bevacizumab played an important role in the treatment of OPG [3, 14]. In addition, MEK (mitogen-activated protein kinase) inhibitor selumetinib, a targeted drug for OPG, is now used in clinical [2, 15]. Whether radiotherapy should be used for the treatment of pediatric OPG is controversial, and the advocates believed that radiotherapy can delay tumor growth effectively, but the opponents argued it would cause long-term vision damage in children. Now, the prevalent view is that radiotherapy should be performed as salvage treatment after chemotherapy or surgical resection. Many papers reported favorable outcomes of local tumor control and VA preservation with radiotherapy [16–18], and they approved to use stereotactic radiotherapy or radiosurgery as the initial treatment for pediatric OPG. Surgery or biopsy is not considered the first choice for pediatric OPG, except for the purpose of histopathological diagnosis. However, for OPG in adults, resection should be the initial treatment to reduce the tumor burden for subsequent radiotherapy or chemotherapy [4].

### 4.2. Outcomes and Prognostic Factor Analysis of OPG

Many prior publications have reported the outcomes and prognostic factors of OPG with different treatments. Fisher et al. documented a total VA preservation rate of 72% after chemotherapy in a multicenter study, the main prognostic factor for VA preservation was tumor site, and there was a poor correlation between radiological findings and VA outcomes [13]; Dodgshun et al. reported a total vision preservation rate of 91% after chemotherapy; the main independent prognostic factors were young age (<2 years) and tumor site (chiasmatic/hypothalamic tumor) [11]; Awdeh et al. treated 20 children diagnosed as OPG with conformal radiation therapy (CRT) and analyzed the data, the total VA preservation rate was 91%, and patients with a history of chemotherapy had a poorer outcome than patients who underwent initial CRT [16]; Combs et al. reported the outcome of 15 OPG patients treated with fractionated stereotactically guided radiotherapy (FSRT), and the 3- and 5-year PFS survival rates were 92% and 72%, respectively, but she did not give the visual outcome [19].

All subjects in this cohort were referral patients from oncology or ophthalmology department; until now, there is no consensus on the treatment of OPG with GKS; the indications we followed are as follows: (1) patients of any VA, with OPG in max diameter ≤ 3cm, with or without chemotherapy/surgical resection history, and (2) patients of any VA, with OPG in max diameter > 3 cm, refuse to or cannot tolerant chemotherapy/surgical resection, with no GKS contraindications. In this cohort, 7 patients had a history of surgical resection, and no patients had prior chemotherapy, because if not necessary, most Chinese parents would resist chemotherapy to their children because of cytotoxicity. The primary goal of GKS was local tumor control, followed by VA preservation. In this study, the 1-, 3-, and 5-year tumor PFS rates were 100%, 92%, and 78%, respectively, and the 1-, 3-, and 5-year VA preservation rates were 92%, 84% and 77%, respectively. There was a moderate correlation between tumor control and VA change. Intratumoral cyst formation and marginal dose were two independent prognostic factors for both tumor control and VA preservation, and intratumoral cyst formation was a risk prognostic factor for both local tumor control and VA preservation, while marginal dose (BED > 60.0 Gy) was a protective prognostic factor for local tumor control, but a risk prognostic factor for VA preservation (BED > 70.0 Gy), so we proposed that marginal dose between 60.0 Gy and 70.0 Gy is optimal for both tumor control and VA preservation. Patients' age, tumor site, and tumor volume were not independent prognostic factors in this study. We observed a higher rate of OS rate of tumor control and VA preservation in pediatric OPG than in adult OPG, but the result was not statistically significant, because the age was not normally distributed in the cohort and the patient number was imbalanced in two subgroups; tumors at different sites showed no different survival rates to irradiation; OARs contributed a higher weight on dose planning than tumor volume.

### 4.3. GKS Treatment Modality

We performed individualized GKS therapies for different OPG patients in recent years. For patients with age > 10 years, tumor located in the orbit, and baseline VA < 0.2, single fraction GKS was usually performed to control tumor growth; otherwise, for patients with baseline VA ≥ 0.2, or tumor located at optic chiasm/hypothalamus, fractionated GKS was usually performed to control tumor growth and preserve the VA; at the same time, fractionated GKS was scheduled in 2-4 fractions and carried out daily with a fractionated marginal dose of 4.5-7.0 Gy (physical dose). In this study, fractionated GKS group provided a higher VA preservation rate than single fraction GKS group, but there is no difference in OS rate for tumor control. Farid Kazemi and colleagues treated 19 OPG patients with various degrees of VA impairment with fractionated GKS; radiation was delivered in 3 fractions with an interval of 12 hours and a fraction physical dose of 6.0 ± 1.2 Gy; during a mean follow-up time of 14 months, patients with low and moderate vision loss at baseline were observed with vision improvement, but there was no significant improvement in patients with severe vision loss at baseline. The results suggested that fractionated GKS can provide good protection for late-responding tissues (such as the optic nerve, chiasm, and hypothalamus) while delivering a high dose to tumors; the result is similar to ours.

### 4.4. Limitation

There were some limitations in this study. First of all, this was a retrospective study; all subjects in this cohort were referral patients from oncology or ophthalmology department and were not representative of the entire OPG population; this was selection bias; the conclusions only suited for a specific patient group, so a randomized, double-blind, and prospective controlled trial is required to achieve a more accurate result. Second, the sample size was not large enough, and there would be deviation in the result because of some outliers; we hope to plan a multicenter study in future to enlarge the sample size and minimize deviation.

## 5. Conclusion

GKS is a safe and effective treatment for OPG; it can be selected as the initial treatment for pediatric OPG that with rapid tumor progression or VA impairment, or as the salvage treatment after chemotherapy or surgical resection, fractionated GKS provides better VA preservation than single fraction GKS in specific patients, and more and more OPG patients will benefit from the individualized GKS treatment.

## Figures and Tables

**Figure 1:** Contrast-enhanced MRI of pediatric OPG before and after single fraction GKS (16.0 Gy). A male OPG patients aged 30 months was observed with proptosis of the right eye, accompanied with VA damage for more than 2 months. (a) MRI at GKS. The tumor is located in the right orbit and surrounded the optic nerve and was homogeneous enhanced on MRI. The baseline VA was 0.15 on the right. (b) Three years after GKS, the tumor volume was smaller than baseline, there was intratumoral necrosis and cyst formation, and tumor enhancement effect declined. The VA remained 0.15, and the proptosis improved significantly. (c) Five years after GKS, the tumor volume remained stable, and tumor enhancement effect declined continuously. The VA was less than 0.1.

**Figure 2:** K-M curve of risk factors for tumor control which were filtered by univariate analysis (log-rank test). Tumor located at the optic chiasm/hypothalamus (a), the existence of intratumoral cyst formation (b), tumor volume > 6 ml (c), and marginal dose (BED) ≤ 60.0 Gy (d) provided a lower survival rate of tumor. The results were statistically significant (*p* value ≤ 0.15).

**Figure 3:** Forest-plot of prognostic factors following multivariate analysis. Among the risk factors, existence of intratumoral cyst formation and marginal dose (BED) were independent prognostic factors for tumor relapse. The results were statistically significant (*p* value ≤ 0.05).

**Figure 4:** K-M curve of risk factors of VA deterioration which were filtered by univariate analysis (log-rank test). Existence of intratumoral cyst formation (a), baseline VA ≤ 0.4 (b), tumor volume > 3 ml (c), and marginal dose (BED) ≥ 70.0 Gy (d) provided a lower survival rate of VA deterioration. The results were statistically significant (*p* value ≤ 0.15).

**Figure 5:** Forest-plot of VA deterioration following multivariate analysis. Among the factors included, existence of intratumoral cyst formation and marginal dose (BED) were independent prognostic factors for VA deterioration. The results were statistically significant (*p* value ≤ 0.05).

**Table 1:** Baseline characteristics of the OPG cohort.

Parameters	*N* = 52
Gender:	
Male	22 (42.3%)
Female	30 (57.7%)
Age (years)	13.8 (2-53)
Diagnosis	
NF1	14 (26.9%)
Sporadic	38 (73.1%)
History of disease (months)	10.4 (1-72)
VA impairment	
No	3 (5.77%)
Yes	49 (94.2%)
Tumor volume (ml)	4.36 (0.25-11.4)
Tumor site	
Hypothalamus/optic chiasm	6 (11.5%)
Intraorbit	46 (88.5%)
Tumor shape:	
Fusiform	42 (80.8%)
Tubular	10 (19.2%)
Surgery history	
No	45 (86.5%)
Yes	7 (13.5%)
Tumor cyst formation	
No	42 (80.8%)
Yes	10 (19.2%)

**Table 2:** Risk factors of local tumor control by uni- and multivariate analyses.

Variable	Univariate analysis		Multivariate analysis	
	HR (confint)	*p* val	HR (confint)	*p* val
Gender	0.83 (0.25-2.74)	0.76		
Age	3.25 (0.7-15.10)	0.17		
Tumor site	0.21 (0.06-0.75)	0.01	0.31 (0.06-1.78)	0.19
Cyst formation	5.77 (1.64-20.29)	0.01	10.1 (1.73-59.08)	0.01
Surgery history	0.26 (0.03-2.03)	0.20		
Tumor volume	5.38 (1.31-22.17)	<0.001	1.43 (1.15-11.11)	0.74
Marginal dose(BED)	0.13 (0.03-0.61)	<0.001	0.11 (0.01-0.87)	0.04

BED: biologically effective dose. *p* val <0.15 suggests statistically significant in univariate analysis. *p* val <0.05 suggests statistically significant in multivariate analysis.

**Table 3:** Risk factors of visual deterioration by uni- and multivariate analyses.

Variable	Univariate analysis		Multivariate analysis	
	HR (confint)	*p* val	HR (confint)	*p* val
Age	1.79 (0.33-9.72)	0.5		
Diagnosis	1.38 (0.26-7.34)	0.7		
Tumor site	1.14 (0.13-9.76)	0.91		
Cyst formation	14.09 (2.27-87.44)	<0.001	46.08 (2.98-713.59)	0.01
VA at baseline	0.86 (0.17-4.26)	0.71	0.2 (0.01-2.789)	0.23
Tumor volume	1.41 (0.25-7.95)	0.87	24.64 (0.6-1019)	0.09
Marginal dose (BED)	3.54 (0.71-17.71)	0.11	239 (3.3-17349)	0.01

BED: biologically effective dose. *p* val <0.15 suggests statistically significant in univariate analysis. *p* val <0.05 suggests statistically significant in multivariate analysis.

## Data Availability

In order to protect the privacy of patients, the data in this study are not open access but are available from the corresponding or first author, for academic reference only.
